RETRACTED

# Curcumin Plant for Colorectal Cancer Prediction and Prevention Using *In Silico* Molecular Analysis; HOT-MELT Extrusion

**DOI:** 10.1155/2022/4376960

**Published:** 2022-06-23

**Authors:** Jamal Moideen Muthu Mohamed, Karuppaiyan Kavitha, Fazil Ahmad, Mohamed El Sherbiny, Doaa Ebrahim, Aida M. EL-Sagheer, Hasnaa Ali Ebrahim, Dalia Mahmoud Abdelmonem Elsherbini, Mosaab Abdella Ebrahim Abdelrahman, Minilu Dejene

**Affiliations:** ^1^College of Pharmacy, Shri Indra Ganesan Institute of Medical Science, Manikandam, Tiruchirapalli 620012, Tamil Nadu, India; ^2^Department of Pharmaceutical Technology, BIT Campus, Anna University, Tiruchirappalli 620024, Tamil Nadu, India; ^3^Department of Anesthesia Technology, College of Applied Medical Sciences, Jubail, Imam Abdulrahman Bin Faisal University, P.O. Box 4030, Jubail, Saudi Arabia; ^4^Department of Basic Medical Sciences, College of Medicine, AlMaarefa University, P.O. Box 1666, Riyadh 11597, Saudi Arabia; ^5^Department of Respiratory Care, College of Applied Medical Sciences, Jubail, Imam Abdulrahman Bin Faisal University, Dammam, Saudi Arabia; ^6^Department of Neuroscience, College of Applied Medical Sciences, Jubail, Imam Abdulrahman Bin Faisal University, Dammam, Saudi Arabia; ^7^Department of Basic Medical Sciences, College of Medicine, Princess Nourah bint Abdulrahman University, P.O. Box 84428, Riyadh 11671, Saudi Arabia; ^8^Department of Clinical Laboratory Sciences, College of Applied Medical Sciences, Jouf University, P.O. Box 2014, Sakaka, Saudi Arabia; ^9^Department of Anatomy, Faculty of Medicine, Mansoura University, Mansoura, Egypt; ^10^Department of Biotechnology, College of Biological and Chemical Engineering, Addis Ababa Science and Technology University, Addis Ababa, Ethiopia

## Abstract

The impact of a soluble complex (SC) of curcumin (CuR) synthesized using hot melt (HM) and hot-melt extrusion (HE) technologies on adenocarcinoma cells for the treatment of colorectal cancer by enhancing CuR solubility is investigated in this work. *In silico* molecular modelling, solubility, drug release, and physicochemical analysis were all part of the phase solubility (PS) study, which featured a novel dyeing test and a central composite design to optimize the best complex (CDD). The optimal HE-SC (1 : 5) enhances solubility (0.8521 ± 0.016 mg·mL^−1^) and dissolution (91.87 ± 0.208% at 30 min), and it has an ideal stability constant (309 and 377 M^−1^) at 25 and 37°C and an A_L_ type of isotherm, implying 1 : 1 stoichiometry according to the findings. An intermolecular hydrogen bond that has not undergone any chemical change and has resulted in the complete conversion of the amorphous form aids in the creation of SC. *In vitro* cytotoxicity was measured at IC_50_ on the SW480 (72 M·mL^−1^) and Caco-2 (40 M·mL^−1^) cells. According to apoptotic studies, apoptosis was responsible for the vast majority of cell death, with necrosis accounting for a small proportion of the total. *In vivo* toxicity was established using a zebrafish model, and a western blot examination revealed apoptosis at the molecular level. It was argued that the novel formulations developed using HE technology are more significant and effective than existing pure CuR formulations.

RETRACTED

## 1. Introduction

Colorectal cancer (CRC) is a tumor that develops in the colon or rectum. It is also known as colon cancer or rectal cancer, depending on the organ involved. CRC is the third leading cause of common cancer in men and the second leading cause of common cancer in women, with the third highest mortality rate of all malignancies globally. CRC is caused by colon polyps, long-term ulcerative colitis, and genetic factors, and it is most commonly diagnosed in people between the ages of 65 and 75. Polyps in the colon are also responsible for cancer cell proliferation, and there are three types of polyps: adenomatous (precancerous), inflammatory polyps, and hyperplastic polyps (cancerous condition). CRC is caused by polyps greater than one centimeter in diameter or the presence of two or more polyps [1, 2]. Dysplasia refers to a form of adenomatous polyp cell that is not cancerous but causes CRC. Cancerous polyps extend to the blood or lymph arteries, lymph nodes, or other organs.

CuR is classed as BCS class-IV because of its limited permeability through the intestinal epithelial cells and poor water solubility (>0.1 mg·mL^−1^ ≈ 111 ng·mL^−1^ at 25°C in aqueous buffer pH) [3]. Despite these advantages, the drug's poor pharmacokinetics, i.e., its low solubility in an aqueous solution, sluggish rate of dissolution, inappropriate digestion in the gastrointestinal system, and poor oral bioavailability, limit its application in human illnesses.

From a pharmaceutical standpoint, it is widely established that drugs that are weakly acidic or basic and poorly water-soluble have poor solubility and bioavailability. Converting the drug's crystalline form to amorphous is a dynamic technique to increase bioavailability, solubility, and dissolution in this scenario. Because crystalline lattices are highly organized, the drugs extreme crystalline structure necessitates greater energy for the dissolving medium to disturb the disordered amorphous form [4]. Amorphous pharmaceuticals have the disadvantage of recrystallizing and becoming thermodynamically unstable. As a result, improving the solubility of insoluble or weakly water-soluble pharmaceuticals is the most difficult challenge in the current drug research in the pharmaceutical industry [5].

RETRACTED

Micronization, nanosizing, the conversion of amorphous form, the enhancement of wettability, prodrugs and salts method, liposomal delivery [6], interaction with a hydrophilic carrier, and solid dispersion technique are just a few of the physicochemical processes that might improve solubility. SC has a wide range of applications as one of the most widely used strategies for improving CuR solubility and dissolution [4].

Briefly, the solid dispersion is a molecularly dispersed drug mix with an inert carrier, such as a hydrophilic carrier. The main strategy, where solid dispersion might increase drug solubility and dissolution, is to convert the crystalline to amorphous form of any drug with smaller particle size for improved wettability [4]. Perhaps, the presence of polymer in the solid dispersion complex promotes stability and inhibits the recrystallization of the drug. Drug-polymer interactions, such as antiplasticization, glass transition temperature, and polymeric carrier viscosity, are among the mechanisms responsible for solid dispersion characteristics [7, 8]. This approach is best suited for drugs that are thermolabile (low melting points).

Breaking the ionic or intermolecular connections in the solute, separating the particles to generate space in the solvent for the solute, and boosting contact between the solvent and the solute ion or molecule are all methods of solubilization. The lipophilic or weakly water-soluble drug is dissolved in an inert carrier, which increases drug solubility and oral bioavailability.

The drug is molecularly distributed into the carrier matrix, resulting in extremely small particles [9], which increases the solid solution carrier dissolving rate. The miscibility (continuous vs discontinuous solid solutions) and molecular distribution of pharmaceuticals contained in the carrier can be used to classify solid solutions (amorphous, substitutional, or interstitial).

Typically, hot melt extrusion (HE) technology is utilized to prepare SC, particularly for pharmaceuticals classified as class II, III, or IV by the Biopharmaceutics Classification System (BCS), which have limited solubility and permeability. HE technology is a continuous process that works under certain conditions that may be tuned for solubility improvement, such as feed rate, rotating screw speed, shear stress, and temperature. Pouring raw materials into a hopper-fed via a heated barrel with a spinning screw that separates into distinct zones achieves mixing and conveyance [10].

Raw materials are fed into a heated barrel with revolving screws that are divided into two mixing and conveying regions. At this moment, the contents begin to change the plasticization process that begins with a melt and then travels the length of the screw barrel [11]. HE technology has the advantages of being a continuous process, having the feature of changing or regulating the release of the drug from the reservoir, having a fast processing time, being easy to scale-up, and requiring no specific solvents.

RETRACTED

As a result of the homogeneous dispersion of drugs and carriers, the generated end products increase bioavailability and dissolution. In addition to SC, the pH modifier in the HE technology effectively changes the pH. It is a promising strategy for enhancing the rate of bioavailability of lipid-soluble drugs (i.e., curcumin) by controlling the rate of release [12]. Stearoyl macrogol-32 glyceride is the chemical name of Gelucire. It is a nonionic surfactant (water-dispersible), mainly used for the lipid-based formulations to increase the solubility and oral bioavailability of the hydrophobic/lipophilic drug [13]. It also acts as a lipid binder during the melting process. GEL has been proved to be safe as determined by toxicological data and is preferred to use in approved pharmaceutical products.

This study used a design with 2 k factorial points extended by 2 k axial points and a center point, where variable numbers are symbolized by the letter 'k. Three or five unique tiers are recommended by these design inputs. The design, however, does not include any of these value groups. CCDs (central composite designs) are fractional factorial or factorial designs with axial (star) points amplified by center points that allow curvature evaluation [14]. The number of star points in a central composite design is always twice as many as the number of components in the plan. For each aspect in the strategy, the star point refers to new outrageous attributes (low and high). It always symbolizes aspects in the design that are worth more than two stars, and it displays both the low and high extreme values for each design component.

## 2. Materials and Methods

### 2.1. Materials, Cell Lines, and Regents

The list of chemicals purchased is as follows: curcumin (CuR; 99% of purity; SRL Pvt. Ltd, Maharashtra, India) and Gelucire 50/13 (GEL) were gift samples from Gattefosse Pvt. Ltd, Mumbai, India. Cell Culture: the colorectal adenocarcinoma cell lines (human) of SW480 and Caco-2 were purchased from NCCS (National Center for Cell Science) in Pune. In DMEM, the cells were seeded (Sigma-Aldrich, USA) and supplemented with FBS (10%), with 20 mL (1%) of streptomycin/penicillin used as an antibiotic (Hi-media, Mumbai, India), at 37°C in a humid atmosphere of 5% CO_2_ in a CO_2_ incubator (Thermo Scientific, USA). Used reagents and chemicals were of analytical grade.

RETRACTED

### 2.2. Phase Solubility (PS) Studies

Higuchi and Connors explain how the PS study has to be carried out [15]. Briefly, this study was carried out by adding an excess quantity of CuR to 25 mL aqueous solutions of different concentrations (1 to 15%) to the GELs solution. The Eppendorf tubes holding the contents were placed in a water bath at a constant temperature (between 25 and 37 ± 0.5°C) for 24 hours, shaking every 30 minutes until the point reached equilibrium. Then, the content was filtered through a Millipore membrane filter (0.45 m), diluted accordingly, and the absorbance was measured using a UV spectrophotometer at 425 nm (Agilent Cary 60, USA). The PS curve may be fabricated using the calculated slope and intercept for the stability complexation constant (K_1:1_). Hence, CuR intrinsic solubility is proportional to the obtained intercept.

(1) $$\begin{array}{c} K\left(1:1\right)=\frac{X}{\left(Y\left(1-X\right)\right)}, \end{array}$$

where *X* and *Y* refer to the slope and intercept, respectively. Also, the enthalpy change (ΔH) determined by the following equation (equation (2)):

(2) $$\begin{array}{c} \ln\frac{K2}{k1}=\Delta H\frac{\left(T2-T1\right)}{kRT1T2}, \end{array}$$

where K1, K2 and T1, T2 refer to the stability constants and difference temperatures in Kelvin of 25 and 37°C, respectively [16]. The change in entropy (ΔS) and Gibbs free energy (ΔG) upon complexation/solubilization were computed from equations (3) and (4), respectively.

(3) $$\begin{array}{c} \Delta G=RT\;\ln\;K, \end{array}$$

where *R* = −8.3144 J·K^−1^·mol^−1^, and K is the gas constant.

(4) $$\begin{array}{c} \Delta S=\Delta H\frac{\left(\Delta H\;-\Delta G\right)}{\left(\Delta G\right)}. \end{array}$$

### 2.3. Molecular Modelling

The BIOVIA discovery studio 2017 (DS) platform was used to assist the molecular interaction experiments employing drug and carriers. The structures were gathered from PubChem and ChemBook databases, converted to a PDB file, and the binding area was defined in a sphere based on the functional group present in the carriers [17]. The grid was, firstly, formed around the bearers of the GEL coordinates of *X* (8.543), Y (0.652), and *Z* (0.043). The top ten best conformations were chosen to investigate CUR-GEL complexation. GEL is docked around CUR, and employing the C-Docker procedure in DS to close with the optimum composite would reduce time for interaction studies. The partnership between drug and carrier complexes was built using the CHARMm developed method.

RETRACTED

### 2.4. Preparation of PM

The physical mixture (PM) of various compositions (1 : 3 to 1 : 7) was physically combined with a mortar and pestle according to the parameters provided by the previous research of Moideen et al. [18] and then screened (# 120; 150–125 m).

#### 2.4.1. Preparation of SC by HM

SC was made by adding CuR to liquefied GEL and stirring continuously at 700 rpm for 15 minutes at 70°C until a homogeneous dispersion was obtained. The liquid solution was quickly cooled to ambient temperature (29°C), then powdered, sieved, and kept in a desiccator at 27°C [17].

#### 2.4.2. Preparation of SC by HE

Using a mortar and pestle, CuR (10% w/w) and GEL (30–70 percent w/w) were well-mixed and milled, and these PM were introduced to the twin screw extruder (CHT20-B, Twin-Screw Extruder, China) at 90°C using a standard configuration as indicated by the supplier [1]. The screw speed was changed from 80 to 120 RPM. Then, using a mortar and pestle, the respective resulting extrusion was crushed into a powder particle and sieved through ^#^120 mesh with a particle size of 150–125 m.

### 2.5. Aqueous Solubility (Solaq) Study

Excess samples (CuR, PM, and SC) were mixed with double-distilled water in 50 mL centrifugal tubes, put in a continuous water bath, and the temperature was maintained at 37 ± 0.5°C for 24 hours, shaking every 30 minutes [19]. Following that, the content was filtered through a Millipore membrane filter (0.45 m), appropriately diluted, and UV absorbance at 425 nm was measured.

### 2.6. Release of CuR in Aqueous Media

The dissolution investigation was carried out in 900 mL of distilled water using a dissolution equipment at 37 ± 0.5°C and 50 rpm, as per Indian Pharmacopoeia specifications (Type II; DS 8000, Lab India, India). Every 5 minutes until 30 minutes, 5 mL of samples was pumped out and filtered using Whatman filter paper (11 *μ*m) at the zeroth time interval. A UV-spectrophotometer set to 425 nm was used to determine the amount of CuR dissolved in the solution. A correction for the fresh dilution was made by replacing the samples with distilled water to preserve the sink condition [16].

### 2.7. Solid State Characteristics

#### 2.7.1. Fourier Transform Infrared Spectrophotometric Analysis (FT-IR)

CuR and excipients were investigated using FT-IR to see whether there was any interaction (structural difference). In an FT-IR spectrophotometer [20] (JASCO/FT-IR-6300, Tokyo, Japan), the IR spectra of solid materials was studied in the solid powder using the KBr disc technique in the wavenumber range of 4000–400 cm^−1^, with a scan speed of 1 cm^−1^.

#### 2.7.2. Powder X-Ray Diffraction Analysis (PXRD)

With the Rigaku Ultima III XRD, the PXRD patterns of samples were studied (Rigaku Co., Ltd., Tokyo, Japan). PXRD was conducted using a Kb filter and Cu Energy at a current of 30 kV and a current of 15 mA. In a prestacked PC software, the samples were successfully spun and inspected at a rate of 1°/min throughout a 2 range of 5–80° (results displayed at 5–40°).

RETRACTED

#### 2.7.3. Differential Scanning Calorimetric (DSC) Analysis

With 3 mg samples positioned in a sealed aluminum pan, the DSC thermogram of powdered materials was detected using a thermal analysis system (DSC; Pyris 6, Diamond TG/DTA; Perkin-Elmer Instruments, Shelton, CT, USA) with an underflow (20 mL·min^−1^) of nitrogen. From 20 to 300°C, the sample was heated at a rate of 10°C·min^−1^. With the pure drug and complexes, the enthalpy changes were computed [21].

### 2.8. Optimization of Ideal Soluble SC Complex

For the less trial preliminaries with second-order trial configurations, the dynamic central composite design (CCD) was adopted. For arithmetical assessment by ANOVA, model equations creation, and response graphs in 3D for each answer, the Design-Expert software® version 11 (Stat-Ease Inc., Minneapolis, USA) was utilized. The quantity of carrier and screw speed (process factors) are independent, whereas aqueous solubility and dissolving time (dependent variables) influence the synthesis of a more soluble SC complex [22].

According to preliminary research, SC made with GEL binary complex using HE technology had higher CuR solubility and dissolution rate than pure CuR and HM-SC. CCD is a dynamic second-order experimental design that consists of 13 trials. The concentration of GEL (*X*_1_) and screw speed (*X*_2_) were tested as independent variables at a two-factor, three-level, with the important quality characteristics Y_1_, aqueous solubility (Solaq; mg·mL^−1^), and Y_2_, released at 5 min (Rel_5 min_; percent), and they were selected as answers.

### 2.9. Dynamic Light Scattering

The determination of hydrodynamic particle size (PS), intensity mean of polydispersity index (PDI), and zeta potential (ZP) of drug and SCs was done through dynamic light scattering technique using Zetasizer [23] (Malvern Instruments Ltd., Nano ZS90, Malvern, UK).

### 2.10. Morphology

The samples were dehydrated without affecting drug decrease by incubation in a series of ethanol (1–5%). Prior to the amplifications at a voltage of 5.0 kV, a thin smear of the samples was gold-coated (100) using a sputter coater. Scanning electron microscope (SEM) pictures were taken with a scanning electron microscope with a zig-zag pattern at a voltage of 5 kv acceleration, according to Carl Zeiss Microscopy Ltd, UK [24].

### 2.11. Dyeing Experiment

A simple new test makes it easier to determine how well a medicine (typically coloured) dissolves in water. Simply put, 10 mg of pure CuR and 60 mg of SCs were dissolved in 15 mL of distilled water, then sonicated for 5 minutes and filtered [25]. White linen (cotton) material pieces of identical size (8 4.5 cm2) were soaked in 50 mL of the aforesaid solution and dried for 1.5 hours. Both the solutions and the dry cloth were photographed.

RETRACTED

### 2.12. MTT Assay

The SW480 and Caco-2 cell lines were used in the MTT (3-(4,5-Dimethylthiazol-2-yl)-2,5-diphenyltetrazolium bromide) test. The cells were grown on 96-well plates, with a cell density of 5 × 10^3^ cells. The DMSO solvent was utilized as a control, using 200 L·well^−1^. Prepared SCs were treated with 20 mL·well^−1^ of MTT reagent (20 mL·well^−1^) and incubated further for 4 hours at 37°C after a 24-hour incubation period. The purple formazan product was dissolved in all of the wells by adding 100 mL of DMSO solvent [26]. Using a plate reader, the aforementioned solution absorption was measured at 570 nm (iMark, Bio-Rad, USA). SC complex concentration required to lower absorbance to half that of the control to obtain the IC_50_ concentration.

### 2.13. Apoptosis Study

The acridine orange and ethidium bromide (AO/EB) twin staining approach was used to investigate apoptosis morphology [27]. SW480 and Caco-2 cells were treated with the estimated IC_50_ concentration of SC complex and incubated for 24 hours before being rinsed with ice-cold phosphate buffer (PBS). The cells were collected in a cluster and diluted with PBS, with a cell density of 5 × 10^5^ cells maintained. On a clean mounted glass slide, the AO/EB twin stain was treated with the aforementioned solution, which included 2.5 M of EB and 3.8 M of AO in PBS. The morphology was studied using a Carl Zeiss fluorescence microscope (Axioscope 2plus, Germany; 400 x magnification) with a 450–490 nm UV filter. A total of 300 cells·sample^−1^ were classified as living, necrotic, or dead, with the nucleus, membrane integrity, and % computed. According to Mohamed et al. [28], Hoechst dye 33258 was also employed to examine the apoptotic morphology of SW480 and Caco-2 cells.

### 2.14. Western Blotting

Western blotting with different polymers was done and published in a prior study [29]. Six-well culture plates contain 1.5 × 106 cells in nutshell. The control and treated cells grew for up to 24 hours at their IC_50_ concentration. The cells were rinsed three times with 0.01 M cold phosphate buffer saline (CPBS) at pH 7.2, and the precipitate was obtained by treating the cells with a CPBS mixture comprising phenylmethylsulfonyl fluoride (100 g·mL^−1^), Tris-base at pH 8.0, NaCl (150 mM), NaNo3 - NP-40 (0.02 percent, 1%), aprotinin (10 M), and Pepstatin A (10 M). The aforementioned mixture was centrifuged (9,000 g) for 5 minutes at 4°C to extract the protein, and the supernatant containing cells was collected for protein assay using a Bio-Rad kit. About 50 g of SDS-PAGE gel (10%) was extracted from the aforesaid combination and processed with a PVDF filter. The proteins were incubated with 10% skimmed milk (SM) in PBST overnight at 4–8˚ C. The filters (membranes) were treated overnight at 4°C with the tested antibodies in SM with PBST after being rinsed with PBS buffer containing 1% Tween 20. After finishing this technique, the proteins were washed three times with TBST before being incubated at room temperature for additional two hours with alkaline phosphatase-conjugated antimouse antibody. Immune complexes were identified from the aforesaid reaction according to the Amersham Bioscience ECL PLUS (chemiluminescence) detection regent standard [30]. The control investigation involved removing a comparable membrane of nitrocellulose and treating it with a 1 : 2000 dilution of actin monoclonal antibody (Sigma) for 2 hours.

RETRACTED

### 2.15. *In Vivo* Zebrafish Toxicity Study

Adult zebrafish (*Danio rerio*) were acquired in the Tamil Nadu district of Tiruchirappalli.

After 3 hours of spawning, healthy eggs, embryos, and larvae were generated. Eggs were obtained and ten healthy embryos were put onto 24-well culture plates containing 1 mL of E3 medium after 3 hpf (hours post-fertilization) [28]. The samples (25–300 *μ*g·mL^−1^) were treated for 96 hours, while the control was kept as placebo. As markers of toxicity, the embryos were checked daily for morphological alterations, hatching, survival rates, edema, spine dislocation, nondepleted yolk, and tail bend.

## 3. Results and Discussion

### 3.1. PS Studies

This research gives key information on the effect of various carriers on CuR solubility. From 25 to 37°C, a typical linear curve in the concentration order ranges from 2.04 × 10^−4^ to 2.12 × 10^−4^ mM. These findings demonstrate an A_L_ type of phase solubility profile (drug solubility rises as a function of carrier concentration) produced by changes in the forces of contact between the drug and the carrier, such as hydrophobic forces and van der Waals forces (Table 1). The PS diagram revealed a slope of less than 1 in GEL, indicating that the complex had 1 : 1 stoichiometry [31]. The slope and intrinsic intercept values of the solubility curves were used to calculate the stability constant (K_1:1_). Plotting the proportion of CuR dissolved versus the GEL concentration (percent w/v) yielded the PS diagram (Figure 1(a)) (See Table 1). The measured value of ΔG was negative, indicating that binding occurs spontaneously (solubilization) and that binding diminishes as the GEL molecular weight increases, and the computed value of ΔH is positive (endothermic). GEL also has high ΔS value (6 KJ·mol·K^−1^), indicating that the complex reaction was endothermic [32].

RETRACTED

Because of additional contacts that allow intermolecular interactions between solvent molecules, the optimal interaction constant is seen at GEL (100 and 112 M^−1^) at 25 and 37°C, respectively. In the range of 100 to 1000 M^−1^, GEL demonstrated the optimal complexation constant. It was thought to influence the solvent interaction with the heteroatom [32]. Apart from CuR's strong solubility in GELs (glycol schemes), the hydrophobic interaction (hydrogen bond) plays a critical role in CuR solubility in the lengthy nonpolar region of GEL and the desirable stable complex because of viscosity.

### 3.2. *In Silico* Interaction

The chosen points of interest of GEL's molecular structure are influenced by computer modeling. The stability of complexes combining drug and ligand molecules was demonstrated and was easy to grasp in *in silico* interaction investigation.  Figure 1(b) illustrates the perfect molecular modeling for the 1 : 1 CuR: GEL complex. An optimal 1 : 1 complex conﬁguration was obtained for CMN with GLR, and the interaction between the complexes showed that CMN hydroxyl group formed two conventional hydrogen bonds with the distance of 2.7 Å, and the ketone group of CMN formed two weak hydrogen bonds with the distance of 2.5 Å, thus, conﬁrming the high tendency of GEL to form the molecular complex obtained from phase solubility study (K_1:1_ = 100, 112 at 25 and 37°C, respectively (Table 1). Subsequently, a complex appears to explain the significant changes in enthalpy (ΔH = 7.2 kJ/mol) and positive changes in entropy (ΔS = 6 J/molK), revealing a stable and soluble complex formed [33]. The minor fluctuations in enthalpy and positive increases in entropy seen in the complex formation, arising from enthalpy-entropy compensation, appear to be clarified by a close-fitting CuR/GEL.

Overall, the nonionic GEL had a superior nonbonded contact with CuR, according to the results of the *in silico* interaction research. These investigations contribute to a deeper knowledge of GEL complexation, and the results are identical to those obtained from PS research. In the SC, the overall perspective on the aqueous solubility of CuR finds that the carrier concentration increases.

### 3.3. Solaq

The Solaq of pure CuR in double-distilled water at 37°C for 24 hours is 0.004 mg·mL^−1^. The solubility of CuR increases by 150 to 180 fold from HE technology and 125 to 148 fold from HM technique in GEL (1 : 3 to 1 : 7), respectively. The Solaq is because of stronger hydrogen bonds between water molecules and an electron-rich oxygen atom in GEL polymer chains. Surface characteristics improve wettability by lowering the liquid (water) surface tension, allowing drug molecules to easily enter into an aqueous environment.

RETRACTED

### 3.4. CuR Release

It causes the powder to float atop the dissolution medium and anticipates contact with the majority of the dissolution medium. It seems that the rate of dissolution of pure CuR was determined to be 1.62% at the end of 30 minutes (double-distilled water). The rate of dissolution on SC with their GEL has a significant burst release (44.12–81.77%) in the first 5–6 minutes, indicating that the complex forms with the GEL or changes to an amorphous/crystal lattice [34]. After 5 minutes, CuR slowly releases from PM and SC in a steady-state manner. The GEL-SC from Figure 2 HE and HM complex reveals that at the end of 30 minutes, 88.21 and 75.55% of CuR was released, respectively, with an initial burst release of 74.91 and 69.17%. In slight dissolution, the pattern of release is because of the metastable supersaturation of CuR in the wet GELs concentration [35].

Apart from nonionic characteristics, viscosity plays an important role in drug dissolution by enhancing the interaction of CuR with the dissolution medium, while the drug is fully dispersed/dissolved in the molten carrier, i.e., the transition from a glassy matrix system to an amorphous form of the drug and the rapid solidification of GEL [36]. In HE technology, hydrophilic GEL carriers successfully convert CuR to amorphous form, resulting in improved drug release. However, with the partial conversion amorphous form of the drug, the result from HM-SCs likely improved drug release.

### 3.5. Solid State Characteristics

#### 3.5.1. FTIR

In the FTIR spectrum of the drug and GELs, CuR reveals a number of characteristic bands representing O-H stretching (alcohol, 3324.68 and 3015.16 cm^−1^), *C*=*O* stretching (1742.37 cm^−1^), *C*=*C* stretching (alkenes: 1629.55 cm^−1^; aromatic: 1597.73 and 1507.1 cm^−1^), C-H bending (1426,1, 1371.14, 960.377, and 810.92 cm^−1^), and stretching vibration [37].

The characteristic bands of GEL show that the peaks at 3269.72, 2915.84, 1730.8, 1465.63, and 719.31 cm^−1^ corresponding to O-H- stretching (alcohol), C-H stretching (SP3), C-O stretching, C-C stretching, and C-H bending vibrations of reduced intensity observed in both SD and PMs associated with CuR have decreased wavelength with PM and SC, implying that the complex has developed through hydrogen bonding. The single peak detected at 2876.31 and 2874.24 cm^−1^ (C-H extending) might be the drug-carrier complexing option site. SC further shows that the N-H expanding band does not emerge at 3343 cm^−1^, implying an intermolecular hydrogen holding between CuR and GEL.

RETRACTED

#### 3.5.2. PXRD

The XRD patterns of CuR show high peaks at 2 of 8.98^o^ and 17.38^o^ (because of the presence of a crystalline drug form) and a succession of small peaks at 23.48, 24.72, 25.68, 26.22, and 27.5^o^ (because of the presence of a crystalline drug form). On contrary, GLR showed amorphous characteristics because of the lack of complete stereo uniformity and presence of the large lateral group in the carrier. PM and SD of CuR-GEL were amorphous with reduced intensity at 2*θ* of 8.98° and 17.38° compared with those of crystalline CMN. The amorphous nature of GEL had been established at SC entirely in their respective diffractogram [38]. The results in GEL show that the amorphous nature is important in both PM and SC because of the reduced intensity, and a significant amount of CuR dissolves in a solid GEL matrix in its amorphous structure, as evidenced by various characteristic peaks of SCs, indicating the transition from a crystalline form of CuR to an amorphous form of SC.

#### 3.5.3. DSC

The endothermic peaks were seen in the DSC curves of CuR (179.8°C) and GEL (49.7°C), which was consistent with previously published results. While CuR interacted with GEL, physiochemical parameters, such as sublimation, melting, and boiling temperatures, altered the thermogram of PM. Because of water molecules freed or entirely transformed to amorphous form or dissolution of the crystalline CuR into the liquid GELs, CuR endothermic peak was completely eliminated in the SC of GEL. In the SC from Figure 3, HM shows a minor peak at about 235°C with lower intensity, which might be related to the melting of CuR at higher temperatures, and it suggests a change in the GEL crystal form [39].

### 3.6. CCD Outcomes on GEL-SC Variables

The coded values for the independent variable GEL concentration (CP) ((1; 300 mg) low value and (+1; 700 mg) high value) and screw speed (SS) ((−1; 80 RPM) low value and (+1; 120 RPM) high value) were determined based on the findings of the first experimental trials.

#### 3.6.1. Sloaq

According to RSM-CCD, the model (quadratic) was significantly suited for the dependent variable [28, 40]. The equation represented by the polynomial equation for response (Sloaq; *Y*_1_) is as follows:

(5) $$\begin{array}{c} Y_{1}=-1.75378+0.002240*A+0.038265*B-0.00625*A*B-0.001*A2-0.000175*B2. \end{array}$$

The model's ability was tested using the sequential lack-of-fit test, F-test, and analysis of variance (ANOVA) findings. For the response *Y*_1_ (*p*=0. 0001), the quadratic predictive model was significant and valid. The *R*^2^ value of 0. 9928 for *Y*_1_ (Solaq) suggests that the experimental and predicted responses (0.9477) are highly correlated [41]. The small CV and adj. *R*^2^ estimates (1.71 and 0.9865, respectively) indicate a good level of precision and dependability in the practical estimation, as well as a large feasible correlation between experimental and projected values.

RETRACTED

The other components and their interactions were not significant (*p* > 0.05). As shown in Figure 4(a), an increase in the quantity of GEL from 300 to 700 mg resulted in a significant improvement in the solubility of CuR from 0.612 to 0.981 mg·mL^−1^, which is dependent on CC (*X*_1_) and SS (*X*_2_) and their Solaq of CuR (Y_1_). This study demonstrates that GEL is capable of effectively resolving the drug's Solaq. The solubility increased, and SS showed a considerable rise in RPM (80 to 120).

#### 3.6.2. Rel_5min_

The following equation represents the polynominal model for response (Rel_5min_; Y2). Equation (6) clearly shows that the independent variables, CP and SS, have positive influence on the response.

(6) $$\begin{array}{c} Y_{2}=+81.66+2.96*A+0.6012*B. \end{array}$$

All independent variables, such as CP and SS, were shown to have a significant progressive influence on Rel_5min_ from 73.11 to 90.47 percent, and it is clear from the positive value for its coefficient that the release improved when CP and SS were increased. The beneficial impact of SS was found to be lower than that of CP. It is also established that the interaction between the independent components is significant [22]. The derived model is significant (F-value = 164.45; *p*=0. 0001), however, the lack of fit is not (F value of 0.1368; *p*=7.88). The differences between the expected (0.9444) and modified (0.9851) *R*^2^ values are visible.

At the end of 5 minutes, the concentration of GEL greatly improves drug release from SC. When GEL concentrations are low, SC release was little. However, when GEL concentrations are increased to 700 mg, a maximum release of up to 90.83 percent may be reached (Figure 4(a), ii). It indicates that raising SS enhanced CuR release rate.

These effects were strongly demonstrated for CPs ranging from 300 to 700 mg, and the center point of SS stated that when SS increased, CuR release rose dramatically, which might be related to 100% amorphization of the drug. The software's final intended solution was used to create an optimal (P14) condition using the answer. To improve technique validation, response variables (Solaq and Rel_5min_) were modified to a maximum range, and the best formulation was found to be 450 mg of GEL and 85 RPM of SS for the manufacture of HE-SC (3 replicates).

RETRACTED

The Solaq (0.8577 ± 0.019 mg·mL^−1^) and Rel_5min_ (90.62 ± 2.302%) experimental values were compared to the predicted values of 0.8387 mg·mL^−1^ and 91.12%, respectively. The prediction error was found to be 0.0131 and 1.51% (Figure 4(a), iii, and iv), respectively, and the low error percentage suggests that the constructed model is optimal and the anticipated outcomes are in strong agreement with the experimental data [28]. The optimized HE-SC complex will be utilized for further study.

### 3.7. SEM

The surface morphologies of pure CuR, GEL (ii), HM-SC (1 : 5) (iii), and optimized HE-SC are supported by the SEM picture in Figure 4(b) (iv). The pure CuR appeared to have a crystalline structure with a typical prism-textured surface and a mean particle size of 15 *μ*m, while GEL appeared to have a smooth surface with an acrystalline-amorphous surface (stereo character). The topological modifications in the HM-SC drug particles partially changed it to amorphous, as demonstrated by a release investigation and a PXRD analysis. As a result of the improved HE-SC, the drug surface seems to be more porous and is seen to be similar and homogeneously disseminated at the molecular level (CuR and GEL morphology were absent). The crystalline CuR was completely transformed into the amorphous form, as seen in the SEM picture.

### 3.8. DLS

In the solution of the PM, the hydrodynamic PS of HM-PM was determined to be 216 ± 9.02 nm with a PDI of 0.254 (Figure 4(c)), revealing a bimodal size distribution (complex including at least two molecules). HE-SC had a hydrodynamic diameter of 152.6 ± 5.9 nm and a PDI of 0.251 (Figure 4(c), ii). ZP is an important parameter for determining the nature of the particle surface and predicting the complex stability (long-term stability). It is a strong argument based on the data from the SEM results [42]. The ZP of HM-SC and HE-SC was found to be -27.4 and -28.7 mV, respectively, indicating that the surface charge was lowered to some extent (Figure 4(c), iii, and iv). As CuR totally converted to an amorphous form, the report indicated a low PDI, suggesting particle size distribution homogeneity, and HE-SC exhibited enough repulsive force to hinder settling or aggregation/agglomeration with long-term storage.

### 3.9. Dyeing Effect

Because of GEL lipophilic nature, pure CuR, HM-SC (1 : 5), and HE-SC (1 : 5) floated on the surface when 10 mg of pure CuR was added to 15 mL of distilled water. In HE-SC, however, the filtrate was clear and transparent, while when HM-SC was added to the same amount of water, it appeared as a solution with yellow hue (Figure 4(d); a ii and iii). The dyeing effects suggest that HE-SC has a high solubilizing capability [15]. This direct functionalized dye test without helpers revealed that HE-SC had a greater coloring influence (Figure 4(d); ii), indicating that the complex solute solubility increased more evenly in water after integration [43].

RETRACTED

### 3.10. MTT Assay

MTT test results show the cytotoxic effects of pure drug and HE-SC on SW480 (Figure 4(e)) and Caco-2 (Figure 4(f)) cell lines. After 24 hours of treatment, the IC_50_ values for SC were 71 (SW480) and 42 (Caco-2 M·mL^−1^), whereas those for pure CuR varied from 147 to 114 M/mL^−1^. The MTT experiment demonstrated that HE and HE-SC had more cytotoxic activity than pure CuR. These findings, according to Manju and Sreenivasan, might be attributable to the effects of cellular uptake profile aberrations, which could contribute to a possible SC effect. The results showed that the SC may transport CuR to SW480 and Caco-2 cells by active targeting through endocytic progression with possible cytotoxicity and HE-SC water solubility [44, 45]. With the increasing concentration of pure CuR and HE-SC, cell viability diminished, although SC had far more potential than native CuR.

### 3.11. AO/EB Staining

The morphology of control or living cells in Figure 5(a) shows that they do not experience apoptotic alterations because they are brilliant green in color and have similar chromatin with an integrated cell membrane. On the other hand, more significant cell death, such as apoptotic and necrotic cells, was detected in labeled cells treated with HE-SC (Figure 5(b)). AO/EB labeling can detect morphological changes during apoptosis, which are critical milestones in cell death [46]. The cytology alterations would have been studied using EB/AO staining had the cells experienced a specific cell death pattern. The cells may be classified into the following kinds based on their fluorescence emission and chromatin geologies: viable cells—have uniform and sorted out structures with green fluorescing cores (Figure 5(a); I), early apoptotic cells—have intact membranes with green fluorescing cores, however, DNA fragmentation has begun, and chromatin buildup is perinuclear and visible in green spindles or patches (Figure 5(a); ii and ii), and late apoptotic cells—have fused or divided chromatin with orange to red fluorescing nuclei with the presence of chromatin cleavage (Figure 5(a); ii and iii) [47]. These outcomes indicates that HE-SC complex could be treated as a lead cell death through apoptosis and little necrosis.

### 3.12. Hoechst 33528 Staining

The cytological alterations in SW480 and Caco-2 cells were seen after 24 hours of incubation, and the physical counting of living, apoptotic, and necrotic cell rates was done using blue Hoechst staining in SW480 and Caco-2 cells, as shown in Figure 5(c). In cells treated with HE-SC rather than pure CuR, more apoptotic cells were seen in both SW480 and Caco-2 cells, with the least number of necrotic cells (Figure 5(d)). Hoechst staining feature demonstrates the ability to identify changes in cell cytology, with a unique pattern of cytoplasm and cell nuclei at a considerable level, detecting cell death [48]. The early apoptotic summary, which included cell shrinkage, expanded chromatin, and cell and nucleus breakdown, as well as a small percentage of necrotic cells, was clearly visible in the HE-SC treated cells.

RETRACTED

### 3.13. Apoptotic Pathway Induced by HE-SC

The western blot confirmed significant variation in the concentration of protein, which reflects the level of apoptosis. Pure CuR and HE-SC-treated cells could effectively destroy the colorectal cells by triggering the caspase pathway in SW480 and Caco-2 cells. The analysis of the cell cycle showed that HE-SC exerts strong cytotoxic action [49]. The protein cyclin D1 plays a large role in cell proliferation by altering the cell signaling pathways by regulating the cell environment. The CUR-treated cells of SW480 and Caco-2 cell lines exhibited extremely reduced cyclin D1 protein levels, thus leading to the elevated number of CRC tumors. The result shown in Figure 6(a) indicates that HE-SC significantly delayed the uptake of cyclin D1, and its potency was greatly reduced. In contrast, cyclin *E* was expressed when compared with pure CuR-treated cells. Tumor suppressing proteins, such as CDK-4, CDK-6, CDK-2, and Rb (Retinoblastoma), were detected during apoptosis in treated samples. The antiapoptotic expression was also observed from the treated cells of HE-SC with CDK-6, and the expression of CDK-4 and CDK-2 was significantly reduced in SW480 and Caco-2 cells. The outcome of the above blotting study shows that CDK inhibits the replication of actin and HCC, which is used for the loading control, and its expression was similar in all lanes in the blot.

Figure 6(a) illustrates the upregulation of protein. The Bax and BCL-2 proteins are, respectively, proapoptotic and antiapoptotic members of the BCL family. The pattern of cell death could be mediated by the caspase family, by the progression of heterodimers between the caspases of proapoptotic and antiapoptotic proteins of BCL-2 protein activation [50]. Remarkably, the outcome of apoptosis is primarily because of the ratio of BCL-2 and BAX, rather than on the quantity of BCL-2 alone.  Figure 6(b) shows the effect of the downregulation of BCL-2 and upregulation of BAX protein on SW480 and Caco-2 cells. In connection with BAX and caspase family, P53 is directly expressed and induces cell cycle arrest (Figure 6(b)), and the prepared HE-SC could trigger P53 by suppressing CRC. The soluble CuR induces cysteine acid proteases belonging to the caspase family in the dynamic proteins for apoptotic enhancer.  Figure 6(b) reveals the induced erosion of the band corresponding to caspase 9 and caspase 3 after treating with soluble CuR (HE-SC). Likewise, PARP (cleaved type) exposed cell destruction as a marker of apoptosis [51]. Moreover, after treating with HE-SC, PARP proteins were cleaved into two parts. Based on the results of the western blot test, prepared HE-SC could be potentially treated for CRC as it significantly enhanced PARP, caspase-3, and caspase -9 proteins.

RETRACTED

### 3.14. Toxicity of HE-SC in Zebra Fish Embryos

Zebra fish embryos are recommended by Kim et al. (2013) as a viable model for new toxicity studies [52]. The proportion of embryos that perished by 96 hours is the mortality rate, and it was compared to the levels in the control group. The levels of death and survival of embryos exposed to various concentrations (25–300 *μ*g/mL) are shown in Figure 6(c). Under a compound stereo microscope, the HE-SC-treated embryos were examined for abnormalities/malformations, such as pigmentation, tail bend, pericardial edema, nondepleted yolk, malformed spine, and distortion of the pericardial sac of the larvae [53]. HE-SC-treated zebrafish egg embryos showed no substantial interruption in their normal development, and the % survivability of larvae showed no significant harm (Figure 6(d)). As a result of the zebrafish toxicity investigation, HE-SC appears to be a promising candidate for innovative drug delivery systems and biomedical engineering.

## 4. Conclusion

This work followed the trend of evaluating the anticancer efficacy of soluble CuR on human colorectal adenocarcinoma cells by examining the effect of HE, and HE technology was applied to increase the solubility and dissolution of CuR. The complex solubility/stability was determined by a phase solubility and molecular modeling interaction of complexes using GELs, which resulted in a better SC complex. Curcumin solubility was increased by 220 times compared to pure curcumin, and a unique dyeing test was conducted for the first time using the complex of curcumin, indicating that its solubility is optimum from HE-SC rather than HM-SC. There are consequences for the reduced particle size produced by HE-SC because of the formation of a suitable complex during the extraction process. Because of the enhanced solubility, it was helpful to the product's overall physicochemical qualities and biological testing. HE-SC is a suitable and prospective preparation for the treatment of colorectal cancer, according to the IC50 concentration, molecular apoptosis by western blot analysis, and *in vivo* toxicity research validated by the zebrafish model. This study showed that obtaining a soluble drug with increased anticancer potential while eliminating toxicity might be a helpful and unique way for the implementation of valuable cancer treatment. This composition, which would be developed in the future using nanotechnology and other unique targeted technologies, would certainly be a novel medicament for public health.

RETRACTED

## Figures and Tables

**Figure 1:** (a) Phase solubility curve of CuR in Milli Q water at 25 and 37°C in the presence of GEL. (b) (A) Molecular modeling for the 1 : 1 complex of CuR: GEL; 2D illustration of a diketo form of CMN showing hydrogen bonding of phenolic OH group. (B) 3D representation of the Dock-pose of CMN (green tubes represent the monomer unit of CuR and grey tubes represent GLR, respectively. The dotted lines indicate most important interactions, and the distances are mentioned in Å units).

**Figure 2:** (a) Bar chart represents the solubility of CuR in HE and HM technology from the ratio of 1 : 3 to 1 : 7. (b) Dissolution release of CuR from PM, HE, and HM-SC (mean ± SD, *n* = 3).

**Figure 3:** (a) The FTIR spectrum, (b) PXRD pattern, and (c) DSC thermogram of pure CuR, GEL, HM-, and HE-GEL.

**Figure 4:** (a) 3D response surface from CCD. (b) Plot of predicted versus actual response of (i) Solaq (mg.mL^−1^) and (ii) Rel_5min_ (%) results from HE-GEL SC. (c) SEM image of (i) Pure CuR, (ii) GEL, (iii) HM-GEL, and (iv) HE-GEL. (D) DLS study: the particle size of (i) CuR-PM and (ii) CuR-SC, and the ZP of (iii) HM-GEL and (iv) HE-GEL. (d) Photograph of (a) solution and (b) immersed cotton clothes of (i) pure CuR, (ii) HE-GEL, and (iii) HM-GEL. *In vitro* cytotoxic outcome of (e) SW480 and (f) Caco-2 cells lines of control, pure CuR, and HE-GEL (Mean ± SD, *n* = 3).

**Figure 5:** Apoptotic fluorescing image of (a) AO/EB and (c) Hoechst 33258 staining observed under fluorescent microscope with SW480 and Caco-2 cells; (i) control; (ii) pure CuR; (iii) HE-GEL. % of live, apoptotic, and necrotic cells of (b) AO/EB and (c) Hoechst 33258 staining after 24 h treatment with SW480 and Caco-2 cells. The significant differences associated with the control are represented by ^*∗∗∗*^*p* < 0.001 and ^*∗∗*^*p* < 0.05, and both are evaluated by student's *t*-test.

**Figure 6:** Western blot represents the number of protein expression in apoptotic lanes after treating with test samples. Lane 1: control, Lane 2: pure CuR, Lane 3: HE-GEL on (a) SW480 and (b) Caco-2 cells. The in vivo toxicity studies of (c) photograph of the zebraﬁsh larvae treated with various concentrations of HE-GEL. (d) Graph representing the viable larvae (%) treated with pure CuR and HE-GEL for 96 hpf. Signiﬁcant differences associated with the control are specified by ^*∗∗∗*^*p* < 0.005 and are calculated with student's *t*-test.

RETRACTED

**Table 1:** Thermodynamic parameters of CuR with GELs at 25 and 37°C (mean ± SD, *n* = 3).

Carrier	T (°C)	Intercept (Mm)	Ka (M^−1^)	ΔG (kJ·mol^−1^)	ΔH (kJ·mol^−1^)	ΔS (kJ·molK^−1^)
GEL	25	2.04^*∗*^10–4	0.01998	100.14 ± 6.17	7.20 ± 0.875	0.06245 ± 0.006
	37	2.12^*∗*^10–4	0.02317	112.05 ± 7.12		

## Data Availability

The datasets used and/or analyzed during the current study are available from the corresponding author on reasonable request.
